The article "Review on Security Issues and Applications of Trust Mechanism in Wireless Sensor Networks" was published in 2022. Journal: Comput Intell Neurosci.

# Review on Security Issues and Applications of Trust Mechanism in Wireless Sensor Networks

**DOI:** 10.1155/2022/3449428

**Published:** 2022-09-27

**Authors:** Zhengxin Xia, Zhe Wei, Huan Zhang

**Affiliations:** ^1^College of Continuing Education, Nanjing University of Posts and Telecommunications, Nanjing 210042, China; ^2^Engineering Research Center of Medicine Information, Nanjing University of Posts and Telecommunications, Nanjing 210042, China; ^3^School of Computer Science, Civil Aviation Flight University of China, Guanghan 618307, China

## Abstract

The scale of wireless sensor networks changes depending on specific application tasks. How to design a relatively simple security mechanism that can extend with the expansion of network scale is an arduous task. As the wireless sensor network mostly adopts the decentralized organization form, once the network nodes are distributed adequately, it is difficult to find out the failure of any node. In addition, the node has weak resistance to physical damage, so any node in the network may potentially become a cause of security vulnerability. In this study, firstly, the security standards that wireless sensor networks should have and the current security challenges faced by the network are discussed in detail, and the importance of security issues in wireless sensor networks is pointed out. Secondly, this paper studies and analyzes the current situation of wireless sensor network security problems including the internal and external attacks and the active and passive attacks. Thirdly, this paper also discusses the significance, concept, and characteristics of reputation and trust, the division and composition of reputation and trust system, and the common applications of the reputation and trust mechanism in wireless sensor networks.

## 1. Introduction

The objects processed by computer systems are mainly abstract things, and these systems do not have insight into the real physical world. Sensors are able to measure the physical quantities such as temperature, pressure, light wave, velocity, electromagnetic wave, and so on and convert the measurement results into electronic signals. Therefore, for computer systems or computable devices, sensors build a bridge from the abstract world to the real world so that the former can obtain almost all kinds of physical information in the real world. However, different from the traditional wired networks, wireless sensor networks, or WSNs, we usually do not need centralized management or fixed infrastructure such as base station and access point. Sensor nodes form the network automatically, and the network cost is relatively low. Therefore, WSNs can be used in situations where there is no infrastructure, or for security reasons, the existing infrastructure does not meet certain conditions. Although WSNs are widely used, security and reliability should be the prerequisite for these applications.

The article "Review on Security Issues and Applications of Trust Mechanism in Wireless Sensor Networks" was published in 2022. Journal: Comput Intell Neurosci.

In this study, firstly, the security standards that wireless sensor networks should have and the current security challenges are discussed in detail, and the importance of security issues in wireless sensor networks is pointed out. Besides, it is of vital importance to develop new security technologies or modify existing security technologies for wireless sensor networks because some traditional security technologies cannot run directly on the network nodes due to their relatively complex algorithms. Secondly, this paper studies and analyzes the current situation of wireless sensor network security problems including the internal and external attacks and the active and passive attacks. Thirdly, this paper also discusses the significance, concept, and characteristics of reputation and trust, the division and composition of reputation and trust system, and the common applications of the reputation and trust mechanism in wireless sensor networks.

## 2. Security Standards and Challenges

In any computer-related environment, security is considered as a nonfunctional requirement, which is not only used to maintain the availability and reliability of the whole system but also related to the protection of information and system. However, in wireless sensor networks, security issues are particularly important because on the one hand, the hardware functions of network nodes are seriously limited, and it is necessary to provide sufficient protection to protect them from malicious attacks; on the other hand, the deployment environment of wireless sensor networks makes it easy for the enemy to obtain sensor nodes illegally and destroy them [1–4]. Any destruction and interference to nodes will have a certain impact on the information obtained in the real world. It is due to the above reasons that WSNs security objectives should have the following standards [5–8], which is shown in Figure 1.

 
*Confidentiality*. Confidentiality generally refers to that unauthorized users cannot obtain confidential or sensitive information, such as network routing information, topology information, and node geographic location information. In wireless sensor networks, confidentiality provides a basic security service for the important data transmitted between network nodes. Confidentiality also ensures that the nodes cannot be eavesdropped or tampered by the third party during data transmission. In the specific implementation process, confidentiality is generally achieved by the secret key mechanism; that is, data packets are encrypted at the sender and decrypted at the receiver. Without the relevant secret key, it is difficult for attackers to access the encrypted information. In addition, it should be pointed out that the data transmitted between nodes does not need to be encrypted. For example, only the data part in the packet is encrypted during data transmission, while in other applications, only the header of the packet is encrypted to protect the identity information of nodes.
 
*Availability*. Availability ensures that network services exist for authorized users; that is, when authorized users need to use some network services, these services exist and are available. In wireless sensor networks, on the one hand, data availability ensures that all nodes submit data to the base station on time, and whenever necessary, the whole network can provide relevant services. In addition, the availability also ensures that nodes are safe and available in the presence of certain attacks.
 
*Integrity*. Integrity makes the data in the whole path between the sender and the receiver without being changed by the enemy [9]. In wireless sensor networks, the integrity of data is particularly important because the nodes are often exposed and unattended, and the communication channel between nodes is also open. Therefore, the transmitted data are easy to be interfered by the enemy channel making the integrity of the data changed.
 
*Authentication*. Authentication enables one party to ensure the legal identity of the other party with whom to communicate, that is, to ensure that the other party is not illegal or fake. In wireless sensor networks, authentication makes the sensing data obtained by the network to come from reliable information sources, and authentication also ensures the reliable identity of communication nodes in the network. In the actual operation of the network, each node should check whether the data it receives come from the real sender.
 
*Data Freshness*. Data freshness ensures that the sensing data sent by nodes in wireless sensor networks is up to date rather than out of date. Data freshness also ensures that the data sent by nodes to base stations can reflect the current situation. At the same time, data freshness can also be used to prevent malicious nodes from sending outdated and invalid information [10].
 
*Forward and Backward Secrecy*. Because nodes in the wireless sensor network have certain constraints on energy supply, some nodes will quit the network due to energy exhaustion after working for a certain period of time. At the same time, according to different application scenarios, there might be new nodes in the network. Therefore, it is necessary to prevent the exiting nodes from breaking the confidentiality of the network, and similarly, it is also necessary to prevent nodes that have just joined the network from cracking any previously used confidential information [11].
 
*Access Control and Nonrepudiation*. Only authorized users can access and use the resources and services provided by the network. Generally, the network should specify the member's permission or the permission group to which the member belongs in advance. Nonrepudiation means that the receiving node cannot deny the data packets it has received, and the sending node cannot deny the data packets it has sent.

The article "Review on Security Issues and Applications of Trust Mechanism in Wireless Sensor Networks" was published in 2022. Journal: Comput Intell Neurosci.

The scale of wireless sensor networks will change depending on specific application tasks. How to design a relatively simple security mechanism that can extend with the expansion of network scale is an arduous task. In most cases, it is necessary to find a compromise between the network performance and the of security mechanism. As the wireless sensor network mostly adopts the decentralized organization form, once the network nodes are distributed adequately, it is difficult to monitor the actual working state of each node, and it is difficult to find out the failure of any node. In addition, the node has weak resistance to physical damage, so any node in the network may potentially become a cause of security vulnerability.

## 3. Internal/External and Passive/Active Attacks

In wireless sensor networks, due to the deployment environment and the limited hardware structure, sensor nodes are more vulnerable to the attacks. Wireless sensor network attacks can be divided into external attacks and internal attacks, and internal attacks are the main security risks of the network. This is because the malicious behavior of nodes in the network or network attacks launched by malicious nodes often disturbs and destroys the normal working nodes in the network. If these attacks are not prevented and handled, they will bring great harm to the whole network. In addition, network attacks can be further divided into active attacks and passive attacks, and active attacks are more harmful in ad hoc wireless sensor networks [12]. WSN attacks are shown in Figure 2.

### 3.1. Internal Attacks and External Attacks

In wireless sensor networks, all nodes are cooperative entities. External attackers are isolated from the network and have no access to the network. Generally, the impact of attacks launched by external attackers on the network is limited, but once the attacker captures the internal nodes of the network and destroys them, such as programming the captured nodes again to execute malicious programs or using nodes with more computing and storage capabilities to replace the captured nodes, the attacks become internal attacks. In contrast, the internal attack is more destructive to the network because the internal nodes are often regarded as legitimate nodes. Internal attacks are more difficult to detect and prevent; for example, the captured nodes can steal confidential information from encrypted data, transfer false information, and modify routing data.

The article "Review on Security Issues and Applications of Trust Mechanism in Wireless Sensor Networks" was published in 2022. Journal: Comput Intell Neurosci.

### 3.2. Passive Attacks and Active Attacks

In passive attacks, the attacker's purpose is to eavesdrop on the flowing information in the network without being detected by the system. Through passive participation in network internal activities, attackers can also obtain a large number of data and conduct data analysis to extract key information. However, due to the lack of clues left by passive attackers, it is difficult to be found.

In active attacks, the attacker can make use of the security loopholes in the network protocol to launch a variety of attacks, such as modifying and deleting the data packets in the routing to make the routing protocol unreliable; for example, in the replay attack, the attacker will maliciously resend the valid routing data packets sent before. The direct result is that the data packets are sent to the wrong destination or make invalid loops in the network, which will eventually lead to network congestion.

Further, a successful active attack by an attacker will seriously damage the function of the network and cause the system to make a wrong judgment and decision. In addition, the more serious threat comes from the physical accessibility of nodes in ad wireless sensor networks. After the attacker locates the sensor node through the communication information, it captures the node and then obtains the key information and other encrypted contents of the captured node through a certain way. Once the attacker succeeds, the attacker can use the encrypted information to monitor the network or inject illegal information into the network. In addition, malicious nodes will also take the way of impersonating legitimate nodes for active attacks. However, different from passive attacks, since the attacker actively participates in the internal activities of the network, there will be signs of malicious attacks in the network.

Stealthy attack is the most common active attack in the data fusion of wireless sensor networks. Its purpose is to inject false data into the data fusion process and ultimately change the decision of base station nodes. In ad hoc wireless sensor networks, decision-making is usually based on all the data collected by nodes, so once there is false data injection, the whole decision-making result may be changed [13]. In response to stealthy attack, Ref. [14] uses eyewitness nodes to ensure that all fusion data are valid, while in Ref. [15], statistical methods are used to test the effectiveness of the fusion data.

The article "Review on Security Issues and Applications of Trust Mechanism in Wireless Sensor Networks" was published in 2022. Journal: Comput Intell Neurosci.

## 4. Trust Mechanism

### 4.1. Concept and Definition

In social science, trust can be understood as follows [16–19]: in social networks, trust refers to the behavior that one party voluntarily relies on the other party in a special environment; trust can also be understood as an intention, i.e., one party intentionally relies on the other party.

In the field of computer science, for example, in a routing information request task, the former is the trustor and the latter is the trusted party. When the routing information is successfully transmitted, it is considered to be a node with good behavior, and then its trust value will be increased; on the contrary, when providing wrong routing information, a node is considered as a malicious node, and the corresponding reduced reputation value is applied as a punishment method. In this mechanism, trust is undoubtedly a double-edged sword. On the one hand, it will consume some resources of the system, and on the other hand, it will greatly improve the security of the system.

### 4.2. Division and Composition of Trust

According to the storage and access of reputation information, the reputation and trust system can be divided into centralized system and decentralized/distributed system. Large e-commerce websites such as Amazon mostly adopt the centralized reputation system and store reputation data in the database associated with websites [20]. For wireless sensor networks, although the centralized reputation system has certain advantages, due to the special structure of network and network nodes, the network system often adopts the decentralized reputation system. In wireless sensor networks, the reputation and trust mechanism has the following characteristics:

1. The mechanism of reputation and trust provides incentives for the benign development of node behavior; that is, it makes nodes more responsible for their own behavior
2. The reputation and trust mechanism provides the prediction of the future behavior of nodes, which can assist in decision-making;
3. The reputation and trust mechanism makes the nodes with good behavior avoid cooperating with the nodes that lack trust. The malicious behavior of nodes leads to the low reputation of nodes themselves, which also makes such nodes have no more opportunities to participate in network cooperation;
4. The reputation and trust mechanism is also conducive to the detection of selfish nodes in the network and timely isolation of malicious nodes in the network.

The article "Review on Security Issues and Applications of Trust Mechanism in Wireless Sensor Networks" was published in 2022. Journal: Comput Intell Neurosci.

## 5. Common Applications of Trust

Reputation and trust mechanisms have been widely studied and applied in distributed systems such as ad hoc networks, P2P networks, grid computing, pervasive computing, and e-commerce. In wireless sensor networks, the reputation and trust mechanism can be combined with other network function algorithms to provide better guarantee and service for the network. Specifically, the reputation and trust mechanism can be applied to the following aspects of wireless sensor networks:

### 5.1. Trusted Data Fusion

In order to ensure the reliability and credibility of data fusion in wireless sensor networks, studies in Refs. [21–33] introduced the reputation mechanism into the network data fusion scheme. In order to deal with the potential malicious nodes in the process of data fusion, combined with reputation management and encryption technology, Ref. [21] proposed a trust-based security data fusion method named blind observation. By adapting the order preserved encryption technology and the sigmoid trust model, the blind observation method can distinguish malicious nodes without decrypting the data sent to the base station and checking the data inside. The security and reliability of data fusion can be ensured by this method. However, in ad hoc wireless sensor networks, the captured or attacked nodes still hold network encrypted information, which is not discussed in Ref. [21].

In order to improve the security of data fusion, Ref. [23] proposed a trust-based intranetwork data fusion method. This method uses the tree data fusion structure and a reputation model based on binomial distribution to detect malicious behavior of nodes. In Ref. [23], the reputation measurement of a node is evaluated by the data it sends, its routing behavior, and its availability. In order to achieve the purpose of reliable data fusion, network nodes only send data to the data fusion nodes whose credibility is higher than the specified threshold value for fusion operation. Although this method may provide security for data fusion, it does not discuss whether the qualified data fusion nodes can rotate to balance the energy distribution of nodes. In addition to using the tree data fusion structure, Refs. [24, 25] also use the cluster structure. In Ref. [25], the data from the node are weighted according to the reputation of the corresponding node, and the common node selects the fusion point according to the reputation of the data fusion node.

To obtain high quality sensory data, Ref. [28] proposed an energy efficient data fusion method ETA based on the binomial reputation model. ETA adopts the cluster node topology structure and uses the reputation mechanism to select the nodes that meet the requirements as data fusion nodes. In addition, in order to find the best path from ordinary nodes to data fusion nodes, ETA also takes into account the residual energy of nodes on the path and the availability of links. In this method, each node maintains two reputation tables: the reputation table about the link availability of the neighbor node and the reputation table about the data fusion ability of the neighbor node. ETA assumes that the location of each node and base station are known in advance and that there is no malicious node injecting false data in the network. But ETA also has the following problems: each node in the cluster must send its data to the upstream node designated by the base station node, which will increase the complexity of the network; to determine the availability of the link between nodes, each node must send data to its neighbor nodes, which will bring extra cost to the network.

The article "Review on Security Issues and Applications of Trust Mechanism in Wireless Sensor Networks" was published in 2022. Journal: Comput Intell Neurosci.

RDAs [22] improve the robustness of data fusion by using the reputation mechanism to identify and isolate malicious nodes in the wireless sensor network data fusion algorithm. The nodes in RDAs adopt the cluster structure and distributed-reputation mechanism. Each node keeps the reputation information of other nodes in the cluster locally and shares the reputation information with other nodes in the cluster. RDAs use LEACH as the underlying data fusion protocol and use the reputation model based on binomial distribution as the node reputation evaluation method.

To ensure the reliability and credibility of data transmitted in WSNs, Ref. [29] proposes a trust evaluation model and data fusion mechanism, which is composed of behavioral trust, data trust, and historical trust. The data trust can be obtained by processing the sensor data, and according to the sensing and forwarding behavior of nodes, the behavior trust is computed. Reference [30] proposes a data fusion and transfer learning empowered granular trust mechanism to handle the data reliability. In order to prevent privacy disclosure and task destruction, a dynamic reward and punishment mechanism is designed to encourage honest users and accurately assess user trust. Reference [31] introduces a data fusion trust model based on rational attributes. It relies on different time attributes to identify the trust of available services, and deep machine learning is used to recursively analyze the attributes and uncertainty characteristics of service providers in continuous shared instances to fuse data with less uncertainty. Reference [32] proposes a trust fusion method consistent with the consortium chain to reach consensus and complete self-organized trust decentralized collaborative learning. In this method, consensus candidates will check others' trust level to ensure that they tend to integrate consensus with users with high trust. Reference [33] proposes a lightweight privacy protection trust evaluation scheme, which can fully balance trust evaluation and privacy protection under low cost so as to facilitate distributed data fusion.

The article "Review on Security Issues and Applications of Trust Mechanism in Wireless Sensor Networks" was published in 2022. Journal: Comput Intell Neurosci.

### 5.2. Trusted Routing

In wireless sensor networks, all nodes are not only the sender of data sets but also the routing and transmission of data from third-party nodes. Therefore, how to route data to the destination through the reliable transmission path becomes one of the key problems in the design and operation of wireless sensor networks when some nodes in the network behave abnormally and violate the specified standards.

Most routing protocols in wireless sensor networks only consider how to maintain the path connectivity between the source node and the destination node and use methods such as the shortest path or minimum spanning tree to construct the data path. However, the above methods rarely consider whether the intermediate nodes involved in the path will cooperate with other nodes to complete the routing and transmission of data packets. Therefore, it is reasonable to think that some intermediate nodes for their own interests (such as legitimate nodes do not respond to the route to save their energy and illegal nodes tamper with data or selectively discard packets) do not complete the routing or packet delivery task according to the protocol. If the routing protocol in wireless sensor network does not have a method to identify selfish behavior or malicious behavior of nodes, the established path may contain the above two kinds of nodes. Therefore, the path may be unstable, the reliability and integrity of data transmission cannot be guaranteed, and the efficiency of the whole network is also low [34].

In order to improve the reliability and security of routing protocols in wireless sensor networks and protect the network from the influence of abnormal behaviors of nodes, the reputation system is combined with the routing protocols of wireless sensor networks in Ref. [34], and the abnormal behaviors of nodes are divided into two categories: selfish behaviors and malicious behaviors. Different processing methods are adopted according to different abnormal behaviors of nodes, the reputation mechanism based on Bayesian theory is combined into the network routing protocol, and the reliability of each node is evaluated according to the data packet delivery. Finally, the reliable data routing path is established according to the reliability of the node.

The article "Review on Security Issues and Applications of Trust Mechanism in Wireless Sensor Networks" was published in 2022. Journal: Comput Intell Neurosci.

According to the observation results of data transmission behavior of nodes, Ref. [34] divides sensor nodes into three categories: friendly, selfish, and malicious. The friendly node will submit the received data packets as they are to ensure the integrity of the submitted data; selfish nodes will randomly discard all or part of the data packets due to their own physical conditions, such as lack of power supply energy, overload, and other reasons, so as to maintain their own physical conditions, and selfish nodes will undoubtedly reduce the reliability of the network; the security and integrity of the network system are often reduced by malicious nodes modifying the contents of the received data packets or deliberately routing the data packets to the wrong receivers.

Reference [35] proposes a trust model based on node behavior to deal with malicious nodes in opportunistic routing and forwarding candidate set. By using pruning and filtering mechanisms, it deletes malicious suggestions and uses dynamic weight calculation method to combine direct trust and indirect trust to get the comprehensive trust. In order to resist attacks such as black hole and selective forwarding, Ref. [36] proposes a trust aware secure routing protocol to resist these attacks, in which each node calculates the comprehensive trust value of its neighbors based on the direct trust, the indirect trust, the volatility factor, and the residual energy. Reference [37] proposes an atomic search sunflower optimization method to provide trust based routing. The method is designed by combining sunflower optimization with atomic search optimization and uses multiple trust factors to identify and isolate attacks and optimize network performance. By using the Markov chain prediction model, Ref. [38] proposes a reliability trust evaluation model for secure routing based on the combination of internal states of nodes and external interaction between nodes. By selecting security nodes based on tolerance constants and selecting opportunity nodes from security nodes for routing, Ref. [39] proposes a routing algorithm based on energy aware trust and opportunity, which uses multipath routing technology with the multihop communication mechanism within and between clusters.

### 5.3. Malicious Node Detection

The security threats of wireless sensor networks come not only from external attacks but also from internal attacks of internal nodes. Although traditional security mechanisms such as the encryption mechanism and the authentication mechanism can prevent some external attacks, these security mechanisms are not so effective for attacks launched by internal nodes with abnormal behavior. Reference [40] proposed a malicious node detection mechanism based on the reputation mechanism. This method adopts the reputation model of Bayesian statistical inference and adds the indirect reputation recommendation from the third party. In Ref. [41], the behavior of malicious nodes modifying data packets was identified by every node monitoring each other. By analyzing the signal strength of data readings received by the physical layer of wireless sensor network nodes, Ref. [42] identifies and prevents malicious nodes that send noise to the network and cause channel conflict. Based on the binomial reputation model, Ref. [43] proposed a location aware method for malicious node isolation and deletion in wireless sensor networks.

The article "Review on Security Issues and Applications of Trust Mechanism in Wireless Sensor Networks" was published in 2022. Journal: Comput Intell Neurosci.

In addition, in order to effectively isolate malicious nodes, Ref. [44] introduces the reputation system into the routing protocol. Its basic principle is that any node in the network uses a certain mechanism to monitor its neighbors and evaluates its trust value according to the behavior of the monitored node; when the reputation value of a neighbor node is less than the defined threshold value, the neighbor node will be considered as a suspicious node. In this algorithm, the change of trust value of neighbor nodes only depends on the observer node. Each observer node shares its suspicious node information, so the noncooperative node will be punished soon. However, this method cannot identify the cheating behavior of malicious nodes. It is only a theoretical framework, and no specific and effective reputation evaluation method is given.

To avoid being judged as a malicious node by the reputation system when the reputation value is lower than the predefined reputation threshold value, and finally isolated by the system, some malicious nodes will attack intermittently and maintain good behavior in the period of not launching the attack so as to obtain a good reputation so that their reputation is generally higher than the reputation threshold. In order to solve the above problems, Ref. [45] proposed a malicious node identification method based on node reputation and time series analysis. In this method, malicious suspected nodes with the above characteristics are defined as subaggressiveness nodes. However, this method does not mention which specific reputation model to select nor does it discuss how to combine with the specific reputation model and gives the corresponding test results. It also does not present the specific method of selecting standard time series parameters.

Reference [46] proposes a malicious node detection method based on online learning algorithm. This method first calculates the credibility of each path in the network according to the collected data packets, then models the path reputation obtained through online learning algorithm, and calculates the trust of each node, and detects malicious nodes through the clustering algorithm. The collaboration-based malicious detection mechanism proposed by Ref. [47] includes a data trust module and a reputation calculation module, which ensures honest data communication and reduces the false positive rate of malicious nodes. Reference [48] proposes an effective malicious node detection scheme based on weighted trust, which can detect malicious nodes in clustered wireless sensor networks. By considering the false positive and false negative examples, the node behavior can be truly handled. Reference [49] proposes a method called perceptron based detection, which uses perceptron and K-means method to calculate the trust value of nodes and detect malicious nodes accordingly, and by optimizing the network routing, the detection accuracy is further improved. Reference [50] proposes a blockchain trust model for malicious node detection in wireless sensor networks. It uses the blockchain smart contract, the quadrilateral measurement and the positioning method of wireless sensor network to realize the detection of malicious nodes in the three-dimensional space.

The article "Review on Security Issues and Applications of Trust Mechanism in Wireless Sensor Networks" was published in 2022. Journal: Comput Intell Neurosci.

Some common applications of trust are shown in Table 1.

As the sociologist Niklas Luhmann said, “Trust and integrity are necessary in our life, it makes the various components of society integrate into one.” Reputation and trust are playing an increasingly important role in human society. In addition, in multiagent systems, due to the uncertainty of agent behavior and in order to protect well-behaved entities from malicious entities, reputation and trust mechanism have been widely adopted and used as a social method [51]. However, the reputation and trust mechanism cannot be simply attributed to security issues. Security is used to prevent an entity from foreign invasion, ensure that another entity is designated with the entity, ensure that the sender and receiver of the message are designated entities, and prevent information from being illegally obtained by other entities. In contrast, reputation and trust are complex and diversified issues. Reputation and trust not only play a role in decision-making but also provide powerful tools for the establishment of relationships among entities in the insecure real world [43]. The reputation and trust mechanism has become an important supplementary tool for many types of network security solutions.

## 6. Conclusions

Due to the lack of infrastructure, wireless sensor networks are vulnerable to a variety of attacks. Without adequate security and physical protection, the number and types of applications of wireless sensor networks will be greatly reduced. Therefore, the security problems of wireless sensor networks need to be solved. As an effective supplement to the traditional security mechanism, the reputation and trust mechanism has attracted the attention of scholars and gradually introduced into ad hoc wireless sensor networks. Nowadays, it has obtained extensive theoretical research and application research, such as the selection of trusted routing path, malicious node identification, and so on. The reputation and trust mechanism can effectively encourage nodes to cooperate and take certain measures to punish malicious behavior of nodes, which not only improves the performance of the network but also enhances the security of the network. In this paper, the security standards and security challenges in wireless sensor networks are discussed in detail. In addition, this paper also discusses the background, significance, concept, and characteristics of reputation and trust, the division and composition of reputation system, and the common applications of reputation and trust mechanism in wireless sensor networks.

The article "Review on Security Issues and Applications of Trust Mechanism in Wireless Sensor Networks" was published in 2022. Journal: Comput Intell Neurosci.

## Figures and Tables

**Figure 1:** Security objectives of WSNs.

**Figure 2:** WSN attacks.

**Table 1:** Common applications of trust.

Representative references	Trust data fusion	Trusted routing	Malicious node detection
[21]	×		
[22]	×		
[23]	×		
[24]	×		
[25]	×		
[26]	×		
[27]	×		
[28]	×		
[29]	×		
[30]	×		
[31]	×		
[32]	×		
[33]	×		
[34]		×	
[35]		×	
[36]		×	
[37]		×	
[38]		×	
[39]		×	
[40]			×
[41]			×
[42]			×
[43]			×
[44]			×
[45]			×
[46]			×
[47]			×
[48]			×
[49]			×
[50]			×

## Data Availability

The data used to support the findings of this study are available from the corresponding author upon request.
